RETRACTED

# Study on Collision Detection and Force Feedback Algorithm in Virtual Surgery

**DOI:** 10.1155/2021/6611196

**Published:** 2021-02-09

**Authors:** Yu Zhang, Dan Luo, Jia Li, Jisheng Li

**Affiliations:** School of Mechanical Engineering, Shenyang University of Technology, Shenyang 110870, Liaoning, China

## Abstract

The development of virtual reality technology is expected to solve traditional surgical training. The lack of methods has brought revolutionary advances in technology. The virtual surgery system based on collision detection and force feedback can enable the operator to have stronger interaction, which is an exploration of the feature of touch in virtual reality technology. Reality is an important indicator of the virtual surgical system. This article improves the realism of the system from the visual and tactile senses and uses the surrounding ball collision detection and force feedback algorithms to build a realistic surgical platform. In the virtual surgery training system, the introduction of force feedback greatly improves the sense of presence during virtual surgery interaction. The operator can feel the softness and hardness of different tissues and organs through the force feedback device. Virtual reality is an interdisciplinary comprehensive technology that has been widely used in military, film, medical, and gaming fields. Virtual reality can simulate the objective world and display it visually, making people feel immersive. Virtual surgery provides surgeons with a recyclable surgical practice platform and can help doctors perform preoperative rehearsals and predict the results of surgery. The design of collision detection and force feedback algorithms is a prerequisite to ensure the immersion and transparency of the virtual surgical training system. This article mainly introduces the collision detection and force feedback algorithm research in virtual surgery, with the intention of providing some ideas and directions for the development of virtual surgery. This paper proposes two collision detection algorithms, space decomposition method and hierarchical bounding box method, and three force feedback algorithms including spring mass point algorithm, Runge–Kutta method, and Euler method to construct virtual surgery collision detection and force feedback. *Experiment with the Overall System Architecture*. This paper proves through experimental results that the average collision detection time after the application of the improved collision detection and force feedback algorithm in the virtual surgery system is more than 80.7% less than the traditional method, which greatly improves the detection speed.

## 1. Introduction

At present, traditional surgical training has major limitations. With the rapid development of computer technology and virtual reality technology, a virtual surgical system combining modern medical technology has emerged [1]. The virtual surgery system can not only improve the efficiency and effect of surgery learning and training to a large extent but also perform preoperative planning and rehearsal of rare operations. More advanced force tactile feedback devices are also increasing, providing a hardware foundation for increasing the operator's immersion in the virtual surgery system.

RETRACTED

With virtual surgery technology, medical staff can use simulation equipment to train how to perform surgery in a computer-generated virtual environment. The virtual surgery system can also record and replay the operations of skilled doctors, thereby greatly saving medical training costs and training time, so as to achieve the purpose of quickly improving the skills of learners [2]. The speed and accuracy of the collision detection algorithm are the prerequisites for real-time virtual surgery; the force feedback control algorithm is the key to ensuring system stability. The virtual surgery training system consists of four two-port networks: operator, force feedback device, sample rack, and virtual environment.

Ong CS believes that virtual surgery involves planning and simulation of surgical reconstruction using three-dimensional (3D) modeling based on individual patient data and is enhanced by simulating planned surgical changes (including implanted devices or grafts), which is described in the study. In one case, virtual heart surgery helped determine the optimal catheter size to reconstruct the right ventricular outflow tract. Ong CS used preoperative magnetic resonance imaging data to perform virtual surgery on a young man with a history of tetralogy of Fallot and pulmonary atresia, constructed his heart in 3D, and simulated three different sizes of RV-PA catheters (18, 20, and 22 mm) implants. Ong CS believes that virtual cardiac surgery can predict the ability to implant a catheter of sufficient size to face continuous somatic cell growth and also allow transcatheter pulmonary valve implantation at some future time. This research is more one-sided [3]. Unger B evaluates the increasing importance of tactile devices and fidelity based on the realism of drilling virtual temporal bones. The virtual surgical contact force depends on the fidelity of the tactile device and is transmitted through the robotic arm. Using the same software and equipment hardware may help to achieve a real feeling. Unger B compares the three degrees of freedom with an ear drill custom built according to the standard. Six ear surgeons performed three virtual mastoidectomy operations on the temporal bone surgery simulator. Modifications are made to make it have gravity compensation and the necessary machinery for use with attached ear drills, and the surgeon uses different hardware platforms for dissection in a random order. Tests show that, for each simulated acoustic characteristic, HD2 improvements are favored (*p* ≤ 0.0004). The high cost of this research is not conducive to popularization [4]. George Jr proposed that backside culling is a preprocessing technology for computer graphics that can speed up the rendering of polyhedrons and showed how to modify this technology to reduce collision detection in physics-based simulation and animation systems [5]. For necessary boundary element inspection, at each time step, George Jr determines an a priori surface that cannot be part of the contact between two polyhedrons and can therefore be eliminated. Then in computer graphics technology, the normal vector of the polygon is compared with the view direction. Here, George Jr compares the normal with one or more relative velocity vectors and rejects it when the direction of movement of the face is opposite to the normal vector. This research is not practical [6].

RETRACTED

The innovations of this paper are as follows: (1) propose the spatial decomposition method and hierarchical bounding box method in collision detection; (2) propose the force feedback spring mass point algorithm; (3) construct the virtual surgery collision detection and force feedback system as a whole architecture; (4) design the lower computer control system.

## 2. Collision Detection and Force Feedback Algorithm in Virtual Surgery

### 2.1. Impact Checking

In order to ensure the authenticity of the virtual environment, users must be able to not only visually see the virtual objects in the virtual environment and their performance but also interact with them immersively [7]. This requires that the solid objects in the virtual environment are not penetrating. It is necessary for the virtual reality system to be able to detect these collisions in time, generate corresponding collision responses, and update the scene output in time, otherwise penetration will occur [8]. It is precisely with collision detection that people can avoid such things as people passing through walls. When the real situation occurs, the virtual world adopts the sense of reality [9].

Accurate collision detection plays a very important role in improving the authenticity of the virtual environment and increasing the immersion of the virtual environment [10]. The high complexity and real-time nature of the virtual reality system puts forward higher requirements for collision detection. In the virtual environment, the conflict detection algorithms between the two models are roughly divided into two categories: spatial decomposition and hierarchical boundary volume [11].

RETRACTED

#### 2.1.1. Space Decomposition Method

The space decomposition method divides the entire virtual space into small cells of equal volume and only detects the intersection of geometric objects occupying the same cell or adjacent cells. This method is usually suitable for similar objects flying between obstacles. Collision detection occurs between geometric objects with relatively uniform distribution in such virtual situations and sparse environments [12].

#### 2.1.2. Hierarchical Bounding Box Method

Hierarchical bounding box method is a popular algorithm in collision detection technology in recent years. This method is widely used in other fields, such as ray tracing. Its basic idea is to use slightly larger and simple geometric bodies (called bounding boxes) to approximate complex geometric objects [13]. Only when the simple geometric bodies containing them intersect can two geometric objects intersect, and further steps are needed [14], to determine whether they really intersect. According to the different types of bounding boxes, there are bounding balls, AABB, and OBB [15]. This method only needs to perform a further intersection test on the overlapping part of the bounding boxes, which can greatly reduce the number of bounding boxes participating in the intersection test and improve the efficiency of collision detection [16].

Which collision method is used depends on the requirements of the control system. If the required virtual surgery system only needs the follow-up relationship between the model and the equipment and does not require force feedback, then the node path of the two geometric models of the instrument and the organ can be directly established at this time, by detecting whether the node path collides. Determine the conflict of the model [17, 18]. However, for devices that require force feedback, it is not only necessary to determine whether the model is in a collision state but also to determine a specific collision position, because the magnitude and direction of the feedback force are directly related to the collision position. At this time, the judgment target should be simplified to the following composition: for the polyhedron of the geometric model (Poly), it is necessary to judge whether the instrument collides with the polyhedron node path on the organ and what collision occurs and then extract the corresponding information from the colliding polyhedron [19], to calculate the magnitude of the feedback force. Both methods have their own advantages and disadvantages. The former is easy to judge, but because it is the bounding box of the judged model, it will happen that the actual model does not collide, but the system has already judged the collision. Although the latter has high judgment accuracy, it must be executed every time [20].

RETRACTED

### 2.2. Force Feedback Algorithm

#### 2.2.1. Spring Mass Point Algorithm

By analyzing the dynamic equation of the spring mass point model, its moving mass point satisfies the following differential equation:

(1) $$\begin{array}{c} M\frac{\partial^{2}X}{\partial t^{2}}+D\frac{\partial X}{\partial t}+K_{\left(X\right)}X=f\left(X\right). \end{array}$$

Among them, *M* represents the mass of the mass point, *D* is the damping coefficient, *X* is the space coordinate of the mass point, *K* is the elastic coefficient of the spring, and *t* is the time constant [21]. The solution of the system equations can be transformed into the problem of solving differential equations of discrete mass points, and the approximate solutions that meet the accuracy range are calculated [22]. If there is a unique solution to this equation, let Δ*t* be the unit time, then in any time period of Δ*t*, through the time difference method and the increment method, for each discrete mass point, the differential equation can be transformed into

(2) $$\begin{array}{c} m^{i}\frac{\partial^{2}X^{i}}{\partial t^{2}}=m^{i}\frac{1}{\Delta t^{2}}\left(X_{i+\Delta t}-2X_{i}+X_{i-\Delta t}\right), \end{array}$$

(3) $$\begin{array}{c} d\frac{\partial X^{i}}{\partial t}=d\frac{1}{2\Delta t}\left(X_{t+\Delta t}-X_{t-\Delta t}\right), \end{array}$$

where *m*^*i*^ represents the mass of the *i*-th mass point and *X*^*i*^ is the coordinate position of the *i*-th mass point. Substituting formulae (2) and (3) into (1), we get

(4) $$\begin{array}{c} m^{i}\frac{1}{\Delta t^{2}}\left(X_{t+\Delta t}-2X_{i}+X_{t-\Delta t}\right)+d\frac{1}{2\Delta t}\left(X_{t+\Delta t}-X_{t-\Delta t}\right)\\ =f_{\mathrm{ext}}^{i}\left(X_{i+\Delta t}\right)-f_{k}^{i}\left(X_{i+\Delta t}\right). \end{array}$$

When Δ*t* approaches infinity, *f*_ext_^*i*^(*X*_*i*+Δ*t*_) can be replaced with *f*_ext_^*i*^(*X*_*i*_), and *f*_*k*_^*i*^(*X*_*i*+Δ*t*_) can be replaced with *f*_*k*_^*i*^(*X*_*i*_), then we can get

(5) $$\begin{array}{c} \left(m^{i}\frac{1}{\Delta t^{2}}+d\frac{1}{2\Delta t}\right)X_{t+\Delta t}=f_{\mathrm{ext}}^{i}\left(X_{i}\right)-f_{k}^{i}\left(X_{i}\right)+m^{i}\frac{2}{\Delta t^{2}}X_{i}\\ -\left(m^{i}\frac{1}{\Delta t^{2}}+d\frac{1}{2\Delta t}\right)X_{i-\Delta t}. \end{array}$$

#### 2.2.2. Runge–Kutta Method

The basic idea of the Runge–Kutta method is to perform a weighted average of the calculated prediction slopes in a certain interval to obtain the average slope value [23]. This calculation method has high accuracy. The formula of the Runge–Kutta method is

(6) $$\begin{array}{c} y_{n+1}=y_{n}+\sum_{i=1}^{s}\phi_{i}k_{i},\;i=1,2,\Lambda ,s. \end{array}$$

Sort in ascending powers according to the time unit, and sort out the following formula:

(7) $$\begin{array}{c} X_{n+1}=X_{n}+s_{1}\Delta t+\frac{1}{2!}s_{2}{\left(\Delta t\right)}^{2}+\frac{1}{3!}s_{3}{\left(\Delta t\right)}^{3}+\Lambda . \end{array}$$

It can be seen from the above formula that the solution formula of the Runge–Kutta method has a high degree of similarity with the expansion of the Taylor series. If *y*(*x*) is continuously derivable in the [*x*_0_, *x*] order on *k*+1, it can be expanded by the Taylor series. The following formula exists:

(8) $$\begin{array}{c} y\left(x_{n+1}\right)=y\left(x_{n}\right)+hy^{\prime }\left(x_{n}\right)+\Lambda +\frac{h^{k}}{k!}y^{\left(k\right)}+R_{k},\\ R_{k}=\frac{h^{k+1}}{k+1}y^{k=1}\left(\xi \right)=o\left(h^{k+1}\right). \end{array}$$

RETRACTED

#### 2.2.3. Euler Method

The basic idea of Euler's method is to use the form of forward difference quotient to approximate the reciprocal, and to discretize the dynamic differential equation [24]. The following formula exists at the particle *m*^*i*^:

(9) $$\begin{array}{c} X^{\prime }\left(m^{i}\right)=f\left(X^{i},f_{\mathrm{ext}}^{i}\right), \end{array}$$

(10) $$\begin{array}{c} X_{i}=X\left(m^{i}\right),\;i=1,2,3,\Lambda ,n. \end{array}$$

After the derivative is approximately replaced by the forward difference quotient, we can get

(11) $$\begin{array}{c} \frac{X\left(m^{i}\right)-X\left(m^{i}\right)}{\Delta t}\approx X^{\prime }\left(m^{i}\right)=f\left(X^{i},f_{\mathrm{ext}}^{i}\right). \end{array}$$

In the formula, Δ*t* is the unit time, when *t*=(*n*+1)Δ*t*, the displacement is

(12) $$\begin{array}{c} X_{n+1}^{i}=X_{n}^{i}+\Delta tf\left(X^{i},f_{\mathrm{ext}}^{i}\right). \end{array}$$

Formula (12) is Euler's integral formula. The error generated after approximate substitution by the form of forward difference quotient is expanded by Taylor series.

(13) $$\begin{array}{c} T_{n+1}=f\left(X_{n+1}\right)-f\left(X_{n}\right)-\Delta tf\left(X_{n},f_{ext}^{i}\right)\\ =f\left(X_{n+1}\right)-f\left(X_{n}\right)-\Delta tf^{\prime }\left(X_{n}\right)\\ =\frac{{\left(\Delta t\right)}^{2}}{2}f^{〞}\left(X_{n}\right)+\frac{{\left(\Delta t\right)}^{3}}{6}f^{〞}\left(X_{n}\right)-o\left({\left(\Delta t\right)}^{4}\right)\\ =o\left({\left(\Delta t\right)}^{2}\right). \end{array}$$

The method part of this article uses the above method to study the collision detection and force feedback algorithm in virtual surgery. The specific process is shown in Figure 1.

RETRACTED

## 3. Collision Detection and Force Feedback Algorithm in Virtual Surgery

### 3.1. Construct the Overall Architecture of Virtual Surgery Collision Detection and Force Feedback System

In the virtual surgery simulation system, the operator can interact with objects in the virtual environment in real time through force feedback devices to obtain a sense of reality and immersion. The virtual surgery simulation system is mainly composed of hardware and software [25].

#### 3.1.1. System Hardware Configuration

The hardware part of the virtual surgery simulation system includes a main computer, a monitor, and a force feedback device. The main computer realizes deformation calculation, collision detection calculation, feedback force calculation, graphics drawing, etc.; the display screen is responsible for displaying the graphic information; the force feedback device is the medium for the user to interact with the virtual world and manipulates the virtual object by accepting the user's operating instructions and output force sense information to the user. The following describes the performance parameters of the main hardware main computer and force feedback equipment and the specific tasks that need to be completed [26, 27].

1. *Main Computer*. Since virtual surgery has high requirements for authenticity and real-time performance, the host computer in the virtual simulation system should have fast computing capabilities, strong graphics processing capabilities, high storage capacity, and stable and reliable functions [28].
2. *Force Feedback Equipment*. Virtual surgery can enable users to have real feelings such as vision and touch in a virtual environment, and force feedback devices are tools that provide users with tactile feelings. When the user interacts with the virtual object through the tentacles, he will feel the surface roughness, softness, and hardness of the touched object [29].

#### 3.1.2. System Software Composition

The virtual surgery system developed in this subject is based on the Windows 10 operating system platform and the compilation environment of Visual Stdio 2017 [2016]. The application is implemented in C# and built on the Unity3D game engine. The force feedback device uses Geomagic Touch, based on Unity3D, and the experimental liver is shown in Figure 2.

1. *Unity3d Software Package*. Unity3d is an open-source C++ library developed by Stanford Labs, which mainly includes multiple modules such as object creation module, device connection module, image rendering, and force rendering, and supports three degrees of freedom, six degrees of freedom, and seven degrees of freedom haptic devices [30]. Due to its lightweight and modular architecture, Unity3d can be easily combined with third-party libraries including graphics or dynamic engines. Unity3d supports three file formats including .3DS, .OBJ, and .STL. When modeling in the system, the CT format of the medical image needs to be converted into these three file formats that can be recognized by Unity3d through other software programs [31].
2. *Visual Rendering Tools*. The graphics rendering tools in the virtual simulation system mainly use the OpenGL (Open Graphics Library) program interface. As the underlying graphics library, OpenGL has seven functional modules such as modeling, lighting and material settings, and texture mapping. It defines a cross-programming language and has a professional graphical interface, rich functions, strong portability, and a wide range of applications [32, 33].

RETRACTED

#### 3.1.3. Construction of Virtual Surgery Platform

The construction of the virtual surgery platform mainly includes the force connection between force feedback equipment and the main computer; the execution of algorithms and the calling of modules are mainly realized by programs. Under normal circumstances, the construction of virtual scenes mainly includes five parts of building a virtual environment, adding force feedback equipment, creating virtual objects, force rendering, and visual rendering.

### 3.2. Design Lower Computer Control System

The design scheme of virtual surgical platform combined with collision detection and force feedback is a servo control system design with high-response speed and high control accuracy in terms of control principles. It can complete fast response and precise tracking and positioning and is used as an important control system in mechatronics. In the design of a virtual surgical platform based on force feedback, the controlled quantity (the output of the system) is a feedback control system for mechanical displacement. Its function is to make the output mechanical displacement (or rotation angle) accurately track the input displacement (or rotation angle). At the same time, it interacts with the human body function simulation environment in the virtual environment. Through calculation and logic processing, the force feedback control of the surgical equipment in the real environment is realized, thereby realizing a virtual operation platform based on force feedback. In the design of the virtual surgery platform, the system design will be discussed from the five main links of controller, controlled object, execution link, detection link, and comparison link, in order to achieve precise and rapid follow-up of the surgery. The mechanical and physical platform virtual environment of the virtual surgery system provides high-precision physical platform data sampling and at the same time quickly realizes accurate force feedback from the virtual environment.

RETRACTED

#### 3.2.1. Comparison Link

The comparison link is in the virtual surgery system; the main controller compares the force feedback control signal obtained from the virtual surgery environment of the host computer with the force feedback control signal obtained from the virtual surgery environment of the host computer by collecting the angle signal of the physical platform, thereby obtaining the difference of the control quantity.

#### 3.2.2. Controller

The controller in the virtual surgery system mainly refers to the DSP2812 control platform. After obtaining the differential signal in the comparison link, the controller obtains the PID algorithm to calculate the output signal of the controller through multiple experiments and then realizes the precise force feedback of the virtual surgery system.

#### 3.2.3. Execution Link

The execution link of the virtual surgical platform is a multichannel motor system. In the design, the high-precision geared motor produced by Maxon is selected as the actuator, which not only can achieve high-precision and high-response torque feedback but also has a high compatibility. The compatibility provides a guarantee for the accurate and reliable operation of the system.

#### 3.2.4. Controlled Object

The mechanical parameters of the controlled object include displacement, speed, acceleration, force, and moment.

#### 3.2.5. Detection Link

The main detection object of this system design is the rotation angle change of the multiaxis mechanical system, and two different angle sensors are used to realize the accurate angle signal acquisition of the system. One is an incremental encoder based on a geared motor, combined with the QEP module of DSP2812 to achieve high-precision angle signal acquisition; the other is a high-precision potentiometer type angle sensor, combined with a high-precision AD acquisition module to achieve nonmotor shaft Fast and high-precision angle signal acquisition.

This part of the experiment proposes the above steps to design a virtual surgical collision detection and force feedback system. The specific process is shown in Table 1.

## 4. Collision Detection and Force Feedback Algorithms in Virtual Surgery

### 4.1. Collision Detection Analysis

1. In the experiment, we still use the number of triangles of the same soft object to test the intersection of the mixed level bounding box, the mixed level bounding box with compressed storage, and the mixed level bounding box with parallel computing, record the average detection time, and then analyze and compare the results. The statistics of the specific results are drawn into charts, as shown in Table 2 and Figure 3.
2. From the above data and experimental image analysis, it can be seen that, in a complex scene with large amounts of data, for the intersection test of rigid objects and soft objects, despite the computational efficiency of hybrid-level bounding box acceleration, there are still many improvements for real-time collision detection. Space, after adding spatiotemporal correlation and compression storage technology to the calculation, storing the leaf node in the storage space of the parent node saves nearly half of the storage and reduces the intersection test element according to the correlation of the time point. The calculation time is much shorter than using the combined-level bounding box alone. The average collision detection time of the system is 80.7% less than the traditional method, which improves the detection efficiency.
3. The specific steps of the collision detection accuracy experiment are as follows: the operator holds the tactile manipulator to move the virtual surgical instrument in the virtual environment; the program records the position coordinates of the manipulator terminal position, and if there is a collision, it will record the position coordinates of the collision point, and if not, in the event of a collision, only the largest bounding ball that has not collided will be recorded, and the system will give a sign of whether it has collided; compare the relationship between the terminal position and node coordinates of the manipulator and the sum of the radii of the two to verify whether a collision has indeed occurred, and the collision flag makes a comparison to verify whether the collision detection is accurate. Record the terminal positions of some manipulators and the *x*, *y*, *z* coordinate positions of the nodes, and their respective radius *r* at this time, and draw them into a chart, as shown in Table 3 and Figure 4.

RETRACTED

Compared with the collision trace calculated by the algorithm, the collision detection based on the data is correct. The algorithm is based on octree partitions and adopts a hierarchical surrounding sphere structure. The manipulator first compares with the root node (the largest bounding sphere) and then gradually advances to the leaf node. It can be seen from the experimental data that the collision detection algorithm of the virtual surgery system is accurate and effective and can be better applied to the virtual surgery system.

### 4.2. Analysis of Force Feedback Algorithm

The tactile interaction device of the system platform is a tactile feedback device of Geomagic Touch developed and produced by STI (Sensable Technologies Incorporated) in the United States. The device provides HLAPI for the calculation of tactile feedback force. The Geomagic Touch force feedback device has 6 degrees of freedom and a three-dimensional work space of 160 mm × 120  mm × 70 mm, a spatial resolution of 0.009 mm, and a maximum applied force of 3.3 N. The force feedback device is shown in Figure 5.

Force feedback can provide mechanical interaction for the virtual reality system, allowing users to experience the reaction force generated by the object model under the action of external forces, thereby enhancing the immersion of virtual surgery users. The Geomagic Touch force feedback interaction device used in this article is a high-precision tactile interaction device produced by a technology company in the United States, which can provide a very large working space and feedback force. Geomagic Touch is the most economical and affordable tactile interactive device today. It has a compact appearance, portable design, and freedom of movement. It is responsive and can well implement general interactive operations. The working parameters of Geomagic Touch are shown in Table 4.

1. The magnitude of the damping friction and Coulomb friction of the Geomagic Touch device will vary according to the position of the operator's arm. Calculate the Coulomb friction and damping friction of Geomagic Touch in the *x*, *y*, and *z* directions, and draw them into graphs, as shown in Table 5 and Figure 6.
2. *X* and *y,* respectively, indicate that the manipulator follows the operator to move in the horizontal and vertical directions, and *z* indicates that it moves in the direction perpendicular to the plane composed of *xy*, so that the force feedback device moves back and forth in four different positions. The friction force is considered constant, so that the friction force in the *x* direction can be obtained. Through the ramp force input, the speed response curve is obtained, and the corresponding parameters can be calculated.
3. In order to verify the real-time performance of the improved Euler algorithm used in the system, the single-step execution time of the traditional Euler algorithm, the improved Euler algorithm, and the Runge–Kutta algorithm are now compared, as shown in Table 6 and Figure 7.
4. It can be seen from the graph that, in the three numerical calculation methods of the improved Euler algorithm, the traditional Euler algorithm, and the Runge–Kutta algorithm, as the number of nodes increases, the single-step execution time gradually increases. Among them, the improved Euler method has the shortest single-step execution time and the fastest deformation frame rate. The evaluation of virtual surgery simulation results includes three aspects: visual fidelity, tactile fidelity, and real time. Visual fidelity requires graphics refresh rate not less than 30 HZ, and tactile fidelity requires feedback force refresh rate not less than 300 HZ. The improved Euler method is adopted, the execution time is short, the calculation efficiency is high, and when the number of nodes is large, the deformation frame rate is also greater than 300 HZ, which fully meets the requirements of virtual surgery simulation.
5. According to the feedback information of collision detection, the deformation or penetration depth can be calculated, and the actual size of the feedback force can be calculated according to the physical model. This force has not been corrected, which is not conducive to ensuring the stability of the system. The self-adaptive limiting output force algorithm can estimate the maximum output force at the next sampling moment to ensure a stable state of the system. After the maximum output force of the virtual environment is calculated, the output feedback force needs to be corrected. Excessive output force will cause not only system instability, but also harm to force feedback equipment and even operators. The calculated maximum output force is used as the output limit value of the current haptic manipulator, and the output force is corrected in real time. When the computing power of the virtual model is less than the maximum allowable force at the current moment, the computing power of the virtual model can be directly fed back to the operator through the tactile manipulator. At this time, the fidelity of the system will not be affected; when the computing power of the virtual model is greater than the current maximum allowable force, the system will directly feed back the calculation result to the user. When the maximum allowable force is at the current moment, the computing power of the virtual model cannot be fully output. Because if it is fully output, the haptic interaction system will become active and unstable, and the haptic manipulator will feed back the maximum output force allowed at the current moment to the operator.

RETRACTED

According to the experimental results, the calculated transparency loss in the *x* direction is 19.31%, the transparency loss in the *y* direction is 9.47%, and the transparency loss in the *z* direction is 0.12%. By comparing the images before and after adding the algorithm, it can be found that the algorithm can ensure the stability of the system, and even when the impedance of the virtual environment is unknown, nonlinear, time-varying, stiffness and damping coefficient are large, as shown in Figure 8. In a certain sampling moment, the interactive feedback force is greater than the maximum limit force and the feedback force is reduced to the limit value, which will help the stability of the system to a certain extent but damage the transparency of the system.

## 5. Conclusions

In recent years, medical accidents have occurred frequently, and more and more attention has been paid to the training of surgeons. However, traditional surgical training has many restrictive factors that make it unable to meet actual needs. The development of virtual reality technology is expected to solve traditional surgical training. The lack of methods has brought revolutionary advances in technology. The virtual surgery system based on collision detection and force feedback enables the operator to have stronger interaction, which is an exploration of the feature of touch in virtual reality technology.

This article improves the realism of the system from the visual and tactile senses and uses the surrounding ball collision detection and force feedback algorithms to build a realistic surgery platform. In the virtual surgery training system, the introduction of force feedback greatly improves the sense of presence in the virtual surgery interaction process. The operator can feel the softness and hardness of different tissues and organs through the force feedback device, but this will also bring about system failure. In order to perform more accurate virtual surgery operations, the stability control algorithm is a very important part.

Although the improved model and force feedback deformation algorithm proposed in this paper have achieved good experimental results in the simulation experiment process, the model and algorithm are more suitable for soft tissue with simple biological characteristics, simple topology, and easy modeling. When it is necessary to simulate soft tissue with complex biological characteristics and tissue structure, such as heart, stomach, and blood vessel modeling, more particles and springs are needed, and the computational complexity will become more and more complex, which will affect the overall performance of the system. Due to the diversity and particularity of human soft tissue, there are still many problems that need to be further studied and improved in the complex soft tissue modeling, which requires a lot of human and material resources, which makes the research into a deadlock.

## Figures and Tables

**Figure 1:** Part of the technical flowchart of this method.

**Figure 2:** Liver diagram of simulated surgery experiment.

RETRACTED

**Figure 3:** Average detection time (unit: ms).

**Figure 4:** Collision detection data.

**Figure 5:** Force feedback device.

**Figure 6:** Coulomb friction and damping friction of Geomagic Touch in the *x, y*, and *z* directions.

**Figure 7:** Single-step execution time distribution of different numerical methods.

**Figure 8:** Comparison of feedback force before and after adding algorithm.

**Table 1:** The experimental procedure of this article.

Experiment on collision detection and force feedback algorithm in virtual surgery	Construct the overall architecture of virtual surgery collision detection and force feedback system	1	System hardware configuration
		2	System software composition
		3	Virtual surgery platform construction
	Design lower computer control system	1	Comparison link
		2	Controller
		3	Execution link
		4	Accused
		5	Testing link

**Table 2:** Average detection time (unit: ms).

Frequency	Number of triangle faces of soft object	Number of triangle faces of rigid object	Space decomposition	Hierarchical bounding volumes	Hybrid bounding box algorithm	Hybrid bounding box algorithm for compressed storage
1	61	50	4.15	4.11	4.23	4.09
2	582	50	4.21	4.19	4.31	4.17
3	1317	50	4.39	4.41	4.42	4.39
4	2134	50	5.07	5.13	5.25	5.07
5	4027	50	6.31	6.92	7.04	6.81
6	5172	50	7.01	7.68	7.73	7.44

**Table 3:** Collision detection data.

Frequency	Robot end position				Node location				Collision sign
	*x* (mm)	*y* (mm)	*z* (mm)	*r* (mm)	*x* (mm)	*y* (mm)	*z* (mm)	*r* (mm)	
1	16.17	21.07	22.71	0.05	24.17	23.07	24.37	1.03	No
2	13.41	22.61	23.06	0.05	23.69	22.91	25.11	1.03	Yes
3	15.22	19.87	21.45	0.05	23.14	23.16	25.91	1.03	Yes
4	17.31	21.42	24.81	0.05	24.81	24.81	23.42	1.03	Yes
5	18.97	19.66	25.79	0.05	25.46	26.92	26.71	1.03	No
6	19.08	21.09	24.77	0.05	26.82	25.74	27.08	1.03	Yes

**Table 4:** Geomagic Touch working parameters.

Friction resistance	<0.26 N
Maximum output force	3.3 N
Hardness	*X* > 7.3 lbs/in (1.26 N/mm)
	*Y* > 13.4vlbs/in (2.31 N/mm)
	*Z* > 5.9 lbs/in (1.02 N/mm)
Continuous output	>0.88 N
Inertia	0∼45 g
Feedback force direction	*x*, *y*, *z*
Location detection	*x*, *y*, *z* digital encoder
Interface	IEEE 802.3 ethernet port (USB option)

**Table 5:** Coulomb friction and damping friction of Geomagic Touch in *x*, *y*, and *z* directions.

	*x*			*y*			*z*	
	*f*_*c*_	*f*_*v*_		*f*_*c*_	*f*_*v*_		*f*_*c*_	*f*_*v*_
*x* − 1	0.11	0.19	*y* − 1	0.13	0.19	*z* − 1	0.16	0.24
*x* − 2	0.13	0.21	*y* − 2	0.15	0.25	*z* − 2	0.17	0.26
*x* − 3	0.16	0.23	*y* − 3	0.14	0.23	*z* − 3	0.19	0.27
*x* − 4	0.17	0.22	*y* − 4	0.16	0.24	*z* − 4	0.14	0.23

**Table 6:** Single-step execution time of different numerical methods.

Numerical methods	Prime number	Time (ms)	Frames
Traditional Euler algorithm	4121	9.81	93.25
	1568	7.14	152.41
	487	2.31	332.61

Improved Euler algorithm	4121	0.91	1449.07
	1468	0.58	2680.18
	447	0.11	9241.33

Runge–Kutta algorithm	734	27	21.35
	682	21	31.47

RETRACTED

## Data Availability

The data that support the findings of this study are available from the corresponding author upon reasonable request.
